RETRACTED

# MRI Using Artificial Intelligence Algorithm to Evaluate Concurrent Chemoradiotherapy for Local Recurrence and Distant Metastasis of Cervical Squamous Cell Carcinoma

**DOI:** 10.1155/2022/4449696

**Published:** 2022-07-28

**Authors:** Youyi Wu, Tingting Chen, Yiwei Huang, Yongchou Li, Xiaoyan Wang

**Affiliations:** ^1^Department of Oncology Radiotherapy, The Third Affiliated Hospital of Wenzhou Medical University (Ruian People's Hospital), Ruian, Wenzhou, 325200 Zhejiang, China; ^2^Department of Radiology and Imaging, The Third Affiliated Hospital of Wenzhou Medical University (Ruian People's Hospital), Ruian, Wenzhou, 325200 Zhejiang, China

## Abstract

The aim of this study was to investigate the magnetic resonance imaging (MRI) features of patients with local recurrence and distant metastasis of cervical squamous cell carcinoma before and after concurrent chemoradiotherapy based on artificial intelligence algorithm. In this study, 100 patients with cervical squamous cell carcinoma with local recurrence and distant metastasis who underwent concurrent chemoradiotherapy were collected as the research subjects, and all underwent MRI multisequence imaging scans. At the same time, according to the evaluation criteria of solid tumor efficacy, patients with complete remission were classified into the effective group, and patients with partial remission, progressive disease, and stable disease were classified into the ineffective group. In addition, an image segmentation algorithm based on Balloon Snake model was proposed for MRI image processing, and simulation experiments were carried out. The results showed that the Dice coefficient of the proposed model segmentation of the reconstructed image was significantly higher than that of the level set model and the greedy algorithm, while the running time was the opposite (*P* < 0.05). The lesion volume (38.76 ± 5.34 cm^3^) in the effective group after treatment was significantly smaller than that in the noneffective group (46.33 ± 4.64 cm^3^), and the rate of lesion volume shrinkage (28.71%) was significantly larger than that in the noneffective group (12.49%) (*P* < 0.05). The relative apparent diffusion coefficient (rADC) value and rADC value change rate of the lesion after treatment in the effective group were significantly greater than those in the noneffective group (*P* < 0.05). In summary, the image segmentation and reconstruction algorithm based on Balloon Snake model can not only improve the quality of MRI images but also shorten the processing time and improve the diagnostic efficiency. The volume regression rate and rADC value change rate of cervical squamous cell carcinoma lesion can reflect the early efficacy of concurrent chemoradiotherapy for cervical squamous cell carcinoma and have predictive value.

RETRACTED

## 1. Introduction

Cervical cancer is one of the common malignant tumors of the reproductive system. The main histological type is squamous cell carcinoma, followed by adenocarcinoma. It has the biological characteristics of invasion, growth, and metastasis. It can have metastasis at different sites with blood circulation, lymphatic circulation, and other routes, including metastasis at the liver, lung, bone, and other sites, and may have corresponding symptoms at the metastatic site [1–3]. In general, patients with cervical cancer in the early stage are not different from chronic cervicitis without any symptoms, and with the development of the disease, it may have abnormal vaginal bleeding, increased leucorrhea, vaginal discharge [4]. For patients with early cervical cancer, the commonly used method is total hysterectomy, followed by extensive total hysterectomy and pelvic lymphadenectomy and para-aortic lymphadenectomy or sampling [5–7]. For patients with advanced disease, if the general condition is not suitable for surgery, radiotherapy can be performed for large cervical lesions, as well as pathological examination after surgical treatment. If high-risk factors are found, adjuvant treatment can be carried out by radiotherapy [8]. The main reasons for cervical cancer treatment failure are local recurrence and distant metastasis. According to clinical statistics, about 31% of patients with cervical cancer will experience tumor recurrence after treatment. The treatment is very difficult and the prognosis is very poor. The average survival time is less than seven months. Therefore, it is very important for the diagnosis and treatment of local recurrence and long-term metastasis of cervical cancer [9].

In the past, cervical cytology was generally used for the screening of early cervical cancer, and colposcopy was performed in patients with abnormal cytology and positive HPV DNA detection; cervical biopsy was the gold standard for the diagnosis of cervical cancer [10–12]. In recent years, with the development of imaging technology and medical technology, CT and MRI have also been gradually applied in the diagnosis of cervical cancer. CT is a cross-sectional scan around a certain part of the human body using an accurate X-ray beam together with a sensitive detector, which is characterized by fast scanning time and high-density resolution, but it is radiant and has a poor display effect on soft tissues [13]. MRI is based on the signal differences of protons in different compounds to distinguish different tissues, including tumor tissues from normal tissues, and has been applied to the imaging diagnosis of various systems throughout the body, with the advantages of no radiation, high soft tissue resolution, and multiple parameters, and is suitable for the brain, spinal cord, great vessels of the heart, joint bones, and pelvic cavity [14]. Pötter et al. [15] used MRI to evaluate the efficacy of adaptive brachytherapy in patients with locally advanced cervical cancer and found that MRI-based adaptive brachytherapy provides effective and stable long-term local control in all stages of locally advanced cervical cancer with limited severe morbidity per organ. Image segmentation is a classic problem in computer vision research and a hot topic in the field of medical image processing. Image segmentation is basically based on the knowledge of digital images, topology, mathematics, and other aspects to construct models, such as threshold-based segmentation methods, region-growth-based segmentation methods, watershed algorithms, and active contour models, and the development of machine learning technology makes image processing methods more diverse [16–18]. Therefore, the MRI image segmentation model was constructed with the help of machine learning technology in order to improve the evaluation accuracy for cervical squamous cell carcinoma.

RETRACTED

In summary, the combination of mathematical models and imaging techniques is currently a hot topic in clinical disease evaluation. Therefore, 100 patients with cervical squamous cell carcinoma who received concurrent chemoradiotherapy were selected as the research objects, and all underwent MRI multisequence imaging scans based on the Balloon Snake model image segmentation algorithm. By comparing the imaging characteristics of the patients in the effective group and the noneffective group, the efficacy of concurrent chemoradiotherapy in patients with local recurrence and distant metastasis of cervical squamous cell carcinoma was investigated based on artificial intelligence algorithms.

## 2. Materials and Methods

### 2.1. Study Subjects

A total of 100 patients with cervical squamous cell carcinoma who received concurrent radiotherapy and chemotherapy in hospital from December 2019 to January 2022 were collected as the study subjects, with an average age of 55.17 ± 9.35 years and an age of 35-77 years. This study had been approved by the ethics committee of the hospital, and patients and their families were informed of the situation and signed informed consent.

Inclusion criteria were as follows: patients who have not received radiotherapy or chemotherapy, patients without contraindications to MRI examination, patients diagnosed with cervical squamous cell carcinoma, patients with complete clinical data, and patients with maximum tumor diameter greater than 1 cm.

RETRACTED

Exclusion criteria were as follows: patients with combined mental diseases; patients with a history of pelvic surgery; patients with other tumors; and patients who did not have regular review one month after chemoradiotherapy.

### 2.2. Treatment Method

All patients were treated with external pelvic irradiation+brachytherapy+concurrent platinum-based chemotherapy. External pelvic irradiation was performed using conformal intensity modulated radiation therapy with external pelvic irradiation dose of 40-45 Gy, 1.8-2.0 Gy per time, 20-25 times, 5 times every seven days. In addition, a dose of 5-8 Gy was added to the parametrial residual lesion and 52-58 Gy to the metastatic lymph nodes. Brachytherapy was performed after the end of external pelvic irradiation, with a total dose of about 28.5 Gy, about 5.8 Gy each time, for a total of 6 times. If the patient's tumor invaded more than one-third of the vagina, two additional vaginal plugs were required. On the first day of radiotherapy, concurrent chemotherapy with cisplatin was administered at a dose of approximately 25-30 mg/m^2^, one time every 7 days.

### 2.3. MRI Examination Method

3.0 T magnetic resonance instrument was used with an eight-channel phased array coil. Diet was forbidden for 8 hours before the examination, and anisodamine hydrochloride was given intramuscularly to the patient half an hour before the examination to reduce gastrointestinal peristalsis and electrolyte artifact. During the examination, the patient was in supine position with feet first entry, and conventional MRI, dynamic contrast enhanced magnetic resonance imaging (DCE-MRI), and magnetic resonance diffusion-weighted imaging (DWI) scanning were performed from the upper edge of the ilium to the lower edge of the pubic symphysis. Conventional MRI scan parameters were as follows: T1-weighted imaging (T1WI): time of repetition (TR) = 3,200 ms, time of echo (TE) = 95 ms, slice thickness 5 mm, interslice distance 2.0 mm, field of view 220 mm, and matrix 521 × 521; T2-weighted imaging (T2WI): TR = 800 ms, TE = 23 ms, slice thickness 4.5 mm, interslice distance 2.0 mm, field of view 220 mm, and matrix 156 × 252. DCE-MRI scan parameters were as follows: TR = 4.5 ms, TE = 1.5 ms, slice thickness 4.5 mm, interslice distance 1.5 mm, field of view 156 mm, and matrix 55 × 55. DWI scan parameters were as follows: TR = 7,500 ms, TE = 65 ms, slice thickness 5 mm, interslice distance 1.5 mm, field of view 220 mm, and matrix 132 × 180.

### 2.4. Image Processing

The obtained MRI images were transmitted to the workstation for processing. The maximum vertical diameter, maximum left-right diameter, and maximum anteroposterior diameter of cervical squamous cell carcinoma lesions were measured, and the lesion volume and regression rate of lesion volume were calculated.

(1) $$\begin{array}{c} V*=l_{1}*l_{2}*l_{3}*\frac{1}{6}\pi ,\\ V_{\%}=\frac{V_{0}^{*}-V_{1}^{*}}{V_{0}^{*}}\times 100\%. \end{array}$$

*V*∗ represents the lesion volume; *l*_1_, *l*_2_, and *l*_3_ represent the maximum vertical diameter, maximum left-right diameter, and maximum anteroposterior diameter of lesion; *V*_%_ represents the volume regression rate; *V*_0_^∗^ represents the lesion volume before treatment; and *V*_1_^∗^ represents the lesion volume after treatment.

RETRACTED

The maximum central level and the upper and lower levels of cervical cancer lesions were selected to measure the apparent diffusion coefficient (ADC) value of the lesions and the gluteus maximus muscle, and the relative apparent diffusion coefficient (rADC) value and rADC value change rate of the lesions were calculated.

(2) $$\begin{array}{c} \text{rADC}=\frac{\text{AD}{\text{C}}_{1}}{\text{AD}{\text{C}}_{2}},\\ V_{\text{rADC}}=\frac{\text{rAD}{\text{C}}_{1}-\text{rAD}{\text{C}}_{0}}{\text{rAD}{\text{C}}_{0}}\times 100\%. \end{array}$$

ADC_1_ represents the ADC value of the lesion, ADC_2_ represents the ADC value of gluteus maximus, *V*_rADC_ represents the change rate of rADC of the lesion, rADC_0_ represents the rADC value of the lesion before treatment, and rADC_1_ represents the rADC value after treatment.

### 2.5. Image Segmentation Algorithm Based on Balloon Snake Model

The Balloon Snake model [19] acts on the contour of any area in the image by introducing balloon expansion and contraction, so that all images are within the scope of Snake. The equation of balloon force can be expressed as follows:

(3) $$\begin{array}{c} \overset{⟶}{f}\left(n\right)=\frac{\left(\left(\partial y/\partial n\right)-\left(\partial x/\partial n\right)\right)}{\sqrt{{\left(\partial x/\partial n\right)}^{2}+{\left(\partial y/\partial n\right)}^{2}}}. \end{array}$$

In Equation (3), *n* represents the normalized arc length, and $\overset{⟶}{f}\left(n\right)$ is a force changed according to the change of the curve. Therefore, the external force of the model can be expressed as follows:

(4) $$\begin{array}{c} f_{\text{outside}}=\alpha_{1}\overset{⟶}{f}\left(n\right)-\alpha_{2}\frac{RH_{\text{outside}}}{\left|RH_{\text{outside}}\right|}. \end{array}$$

In Equation (4), −(*ℜH*_outside_/|*ℜH*_outside_|) means the normalized value of Gaussian potential energy, and *α*_1_, *α*_2_ are all weight coefficients. When *α*_1_ > 0, the contour curve will expand outward; when *α*_1_ < 0, the contour curve will contract inward; when |*α*_1_| < |*α*_2_|, the contour curve will not cross the edge. It is assumed that the elastic potential energy is *λ*_1_(*n*) and the rigid parameter is *λ*_2_(*n*); the model can be expressed as follows:

(5) $$\begin{array}{c} T\left(n\right)=\lambda_{1}\left(n\right)+\lambda_{2}\left(n\right)+\alpha_{1}\overset{⟶}{f}\left(n\right)-\alpha_{2}\frac{RH_{\text{outside}}}{\left|RH_{\text{outside}}\right|}. \end{array}$$

The image segmentation process based on the above model can be shown in Figure 1. Firstly, Gaussian fuzzy preprocessing was carried out on the image; then, points were automatically selected on the image to form a circular boundary, and then, automatic sketching was carried out to obtain the optimal image segmentation result by adjusting parameters.

RETRACTED

### 2.6. Image Segmentation Evaluation Indicators

The level set model [20] and greedy algorithm [21] were compared with the proposed model, and the Dice coefficient and average running time per image were counted using the results of manual segmentation by the physician as the gold standard.

(6) $$\begin{array}{c} \text{Dice}=\frac{2\left|P\cap Q\right|}{\left(\left|P\right|+\left|Q\right|\right)}. \end{array}$$

*P* represents the standard result, and *Q* represents the model segmentation result. The value of Dice coefficient is between 0 and 1, which indicates that the image segmentation result is better.

### 2.7. Imaging Evaluation of Clinical Efficacy

According to the response evaluation criteria in solid tumors [22] and in combination with the results of MRI image evaluation, the therapeutic effects of tumors were classified as complete response (complete disappearance of lesions), partial response (the long diameter of lesions after treatment was reduced by more than 30% compared with that before treatment), disease progression (the long diameter of lesions after treatment was increased by more than 20% compared with that before treatment), and stable disease (the long diameter of lesions after treatment was reduced by less than 30% or increased by less than 20% compared with that before treatment). Complete response patients without lymph node metastasis were included in the effective group, and the remaining patients were included in the noneffective group.

The general information of the patients (age, height, weight, maximum tumor diameter, squamous cell carcinoma associated antigen (SCC), and International Federation of Gynecology and Obstetrics (FIGO) staging) was collected.

### 2.8. Statistical Methods

Data were analyzed using SPSS 22.0 statistical software, measurement data were expressed as mean ± standard deviation ($\overset{¯}{x}\pm s$), and enumeration data were expressed as percentage (%). One-way analysis of variance was used for pairwise comparisons. The difference was statistically significant at *P* < 0.05.

RETRACTED

## 3. Results

### 3.1. Segmentation and Reconstruction Effect of Different Models on MRI Images

Figure 2 showed the segmentation and reconstruction effect of different models on MRI images. The Dice coefficient of the proposed model segmentation and reconstruction of image was significantly higher than that of the level set model and greedy algorithm, while the running time was significantly less than that of the level set model and greedy algorithm, and the difference had statistical significance (*P* < 0.05).

Figure 3 showed the image segmentation results of different models. The lesion display of the original image was not clear, and there were many artifacts and noise. After segmentation and reconstruction of the three models, the image quality was significantly improved, while the image sharpness after segmentation and reconstruction of the proposed model was the highest, and the artifacts and noise were significantly reduced.

### 3.2. Efficacy Evaluation Results

Figure 4 suggested that of the 100 patients, 63 had complete response, 28 had partial response, 8 had stable disease, and 1 had disease progression. 10 patients had response or stable disease after treatment but developed lymph node metastasis, including pelvic lymph node metastasis in 6 patients, abdominal aortic lymph node metastasis in 3 patients, and common iliac lymph node metastasis in 1 patient.

### 3.3. Comparison of General Data

Figure 5 showed that the differences of age, height, weight, maximum tumor diameter, and SCC between the effective group and noneffective group were not significantly different (*P* > 0.05). There was significant difference in FIGO stage between the effective group and the noneffective group (*P* < 0.05). The FIGO stage of the effective group was stage IIa in 14 cases (22.22%), stage IIb in 33 cases (52.38%), stage IIIa in 6 cases (9.52%), and stage IIIb in 10 cases (15.87%). FIGO stage of the noneffective group included 5 cases in stage IIa (13.51%), 33 cases in stage IIb (24.32%), 20 cases in stage IIIa (54.05%), and 10 cases in stage IIIb (8.11%).

### 3.4. Case Analysis

The case is a 50-year-old married woman with no previous history of infectious diseases such as hepatitis, tuberculosis, or malaria and denying any history of trauma, blood transfusion, or food allergy. MRI image showed that T1 signal was isointense, similar to the surrounding muscle layers, and of little value for staging. T2 was medium and high signal, unlike intima and hypointense stroma. The lesion can be observed in the sagittal view in the posterior endocervical canal, which was significantly different from the surrounding normal stroma (Figure 6).

RETRACTED

A 63-year-old female patient had no dizziness, vertigo, nausea, vomiting, frequent urination, urgent urination, anal bulge, or other discomforts, denying the history of heart disease, diabetes, and other chronic diseases; denying the history of hepatitis, malaria, tuberculosis, and other infectious diseases; and denying the history of trauma, blood transfusion, or food allergy. MRI image showed low signal intensity on T1WI and high signal intensity on T2WI, and the lesions showed a round mass, thickening of the posterior bladder wall, and dilatation of the distal ureter (Figure 7).

### 3.5. Comparison of Lesion Volume between Two Groups before and after Treatment

There was no significant difference in lesion volume between the effective group and the noneffective group before treatment (*P* > 0.05). After treatment, the lesion volume of the effective group was significantly smaller than that of the noneffective group, and the difference was statistically significant (*P* < 0.05). The lesion volume (38.76 ± 5.34 cm^3^) in the effective group after treatment was significantly smaller than that in the noneffective group (46.33 ± 4.64 cm^3^), and the rate of lesion volume shrinkage (28.71%) was significantly larger than that in the noneffective group (12.49%) (*P* < 0.05), as shown in Figure 8.

### 3.6. Comparison of rADC Value between Two Groups before and after Treatment

There was no statistically significant difference in rADC values of lesions between the effective group and noneffective group before treatment (*P* > 0.05). The rADC value of lesions in patients of the effective group after treatment was significantly higher than that in patients of the noneffective group, and the difference was statistically significant (*P* < 0.05). The change rate of rADC value in the effective group was significantly higher than that in the noneffective group, and the difference was statistically significant (*P* < 0.05) (Figure 9).

## 4. Discussion

As one of the common malignant tumors in women, the incidence of cervical cancer is increasing year by year and tends to be younger, which is a major cause of death in young and middle-aged women. At present, the main clinical treatment methods for cervical cancer are surgical treatment, chemoradiotherapy, and immunotherapy, and physicians need to select the appropriate treatment plan according to the tumor stage [23]. Therefore, 100 patients with cervical squamous cell carcinoma who underwent concurrent chemoradiotherapy in hospital were collected as the study subjects, and MRI multisequence imaging scans were performed. In addition, in order to provide the quality of MRI images, an image segmentation and reconstruction algorithm based on the Balloon Snake model was proposed and compared with the level set model and the greedy algorithm. First, it was found that the Dice coefficient of the proposed model segmentation and reconstruction of image was significantly higher than that of the level set model and the greedy algorithm, while the running time was significantly less than that of the level set model and the greedy algorithm, and the difference was statistically significant (*P* < 0.05), which was similar to the results of Mayadev et al. [24], indicating that the image segmentation and reconstruction algorithm based on Balloon Snake model can not only improve the quality of MRI images but also shorten the processing time and improve the diagnostic efficiency. From the actual segmentation image results, the lesion display of the original image was not clear, and there were a large number of artifacts and noise. After segmentation and reconstruction of the three models, the image quality was significantly improved, while the image sharpness of the proposed model segmentation and reconstruction was the highest, and the artifacts and noise were significantly reduced, which corresponded to the above data results.

RETRACTED

The clinical efficacy of the patients was evaluated according to the response evaluation criteria for solid tumors and the results of MRI image evaluation, and it was found that of the 100 patients, 63 had complete response, 28 had partial response, 8 had stable disease, and 1 had disease progression, and the patients with complete response were classified as the effective group, and the remaining patients were classified as the noneffective group. Comparison of the basic data between the two groups revealed that there were no significant differences in age, height, weight, maximum tumor diameter, and SCC between the effective group and the noneffective group (*P* > 0.05), while there was significant difference in FIGO stage between the effective group and the noneffective group (*P* < 0.05), which indicated that FIGO stage may be correlated with the clinical efficacy of patients. The MRI image characteristics of cervical squamous cell carcinoma showed low signal intensity on T1WI and high signal intensity on T2WI, and the lesion was in the posterior cervical canal in the sagittal view, which was significantly different from the surrounding normal matrix. The lesion volume after treatment in the effective group was significantly smaller than that in the noneffective group, while the regression rate of lesion volume was significantly greater than that in the noneffective group, and the difference was statistically significant (*P* < 0.05). The degree of lesion volume reduction can reflect the clinical efficacy of patients to a certain extent; this is similar to the findings of Chopra et al. [25], showing that the degree of lesion volume regression in patients who responded to concurrent chemoradiotherapy was higher than that in patients who did not respond. The rADC value and change rate of rADC value of the lesion after treatment in the effective group were significantly greater than those in the noneffective group, and the differences were statistically significant (*P* < 0.05), which indicated that the rADC value and change rate of rADC value could reflect the early efficacy of concurrent chemoradiotherapy for cervical squamous cell carcinoma and had predictive value.

RETRACTED

## 5. Conclusion

In this study, 100 patients with cervical squamous cell carcinoma were included as the research objects, and all of them underwent MRI multisequence imaging scans based on the Balloon Snake model. The results found that the image segmentation and reconstruction algorithm based on Balloon Snake model can not only improve the quality of MRI images but also shorten the processing time and improve the diagnostic efficiency. The regression rate of cervical squamous cell carcinoma lesion volume and the change rate of rADC value can reflect the early efficacy of concurrent chemoradiotherapy for cervical squamous cell carcinoma, which had predictive value. However, the size of the included samples is small and the included samples are originated from the same hospital, so the obtained data are not universal, which may have an impact on the results. Moreover, for the long-term prognosis of patients after chemoradiotherapy, no follow-up record is made. In the future, it was necessary to reinclude the study subjects to observe the long-term recovery of patients. In conclusion, it provides a reference for concurrent chemoradiotherapy in patients with cervical squamous cell carcinoma and imaging evaluation of efficacy.

## Figures and Tables

**Figure 1:** Image segmentation flow based on the Balloon Snake model.

**Figure 2:** Segmentation and reconstruction effect of different models on MRI images: (a) Dice coefficient; (b) average running time. ^∗^Compared with the proposed model, *P* < 0.05.

**Figure 3:** Display of image segmentation results by different models: (a) original image; (b) level set model; (c) greedy algorithm; (d) proposed model.

**Figure 4:** Efficacy evaluation results. 1-4: complete response, partial response, stable disease, and disease progression.

RETRACTED

**Figure 5:** Comparison of general data between the effective group and noneffective group of patients: (a) age, height, and weight; (b) maximum tumor diameter; (c) SCC; (d) FIGO stage.

**Figure 6:** MRI image of a female patient. Female, 50 years old, married, admitted with irregular vaginal bleeding for 15 days: (a) T1WI; (b) T2WI; (c) DCE-MRI; (d) DWI.

**Figure 7:** MRI image of a female patient. Female, 63 years old, admitted twice with abnormal vaginal bleeding 10 years after menopause: (a) T1WI; (b) T2WI; (c) DCE-MRI; (d) DWI.

**Figure 8:** Comparison of lesion volume between the two groups before and after treatment: (a) lesion volume; (b) regression rate of lesion volume. ^∗^Compared with the effective group, *P* < 0.05.

**Figure 9:** Comparison of rADC values of lesions between the two groups before and after treatment: (a) rADC value of lesions; (b) change rate of rADC value of lesions. ^∗^Compared with effective group, *P* < 0.05; ^#^Compared with before treatment, *P* < 0.05.

## Data Availability

The data used to support the findings of this study are available from the corresponding author upon request.
